# MiR-590-5p inhibits colorectal cancer angiogenesis and metastasis by regulating nuclear factor 90/vascular endothelial growth factor A axis

**DOI:** 10.1038/cddis.2016.306

**Published:** 2016-10-13

**Authors:** Qingxin Zhou, Yuekun Zhu, Xiaoli Wei, Jianhua Zhou, Liang Chang, Hong Sui, Yu Han, Daxun Piao, Ruihua Sha, Yuxian Bai

**Affiliations:** 1 Department of Gastrointestinal Oncology, The Third Affiliated Hospital, Harbin Medical University, Harbin, China; 2 Department of General Surgery, The First Affiliated Hospital of Harbin Medical University, Harbin, China; 3 Department of Neurosurgery, The Third Affiliated Hospital, Harbin Medical University, Harbin, China; 4 Department of Digestive Disease, Hongqi Hospital, Mudanjiang Medical University, Mudanjiang, China

## Abstract

Altered expression of microRNA-590-5p (miR-590-5p) is involved in tumorigenesis, however, its role in colorectal cancer (CRC) remains to be determined. In this study, we focused on examining the effects of different expression levels of miR-590-5p in cancer cells and normal cells. Results showed that there are lower expression levels of miR-590-5p in human CRC cells and tissues than in normal control cells and tissues. Similarly, in our xenograft mouse model, knockdown of miR-590-5p promoted the progression of CRC. However, an overexpression of miR-590-5p in the mice inhibited angiogenesis, tumor growth, and lung metastasis. Nuclear factor 90 (NF90), a positive regulator of vascular endothelial growth factor (VEGF) mRNA stability and protein synthesis, was shown to be a direct target of miR-590-5p. The overexpression of NF90 restored VEGFA expression and rescued the loss of tumor angiogenesis caused by miR-590-5p. Conversely, the NF90-shRNA attenuated the increased tumor progression caused by the miR-590-5p inhibitor. Clinically, the levels of miR-590-5p were inversely correlated with those of NF90 and VEGFA in CRC tissues. Furthermore, knockdown of NF90 lead to a reduction of pri-miR-590 and an increase of mature miR-590-5p, suggesting a negative feedback loop between miR-590-5p and NF90. Collectively, these data establish miR-590-5p as an anti-onco-miR that inhibits CRC angiogenesis and metastasis through a new mechanism involving NF90/VEGFA signaling axis, highlighting the potential of miR-590-5p as a target for human CRC therapy.

MicroRNAs (miRNAs) are a class of small endogenous noncoding RNAs of 22 or so nucleotides, which negatively regulate gene expression by binding to the 3′-untranslated region (UTR) of their target mRNAs.^1^ It has been shown that miRNAs have critical roles in apoptosis, development, differentiation, cell proliferation, and tumorigenesis.^2, 3^ In addition, recent evidence has indicated that miRNAs can function as oncogenes or tumor suppressors.^4, 5^ Many miRNAs were found to be aberrantly expressed in colorectal cancer (CRC) with the downregulation of miR-601, miR-192, miR-345, miR-215, and miR-612, and the upregulation of miR-223, miR-18a, miR-155, miR-31, and miR-224, when compared with those found in normal colon mucosa.^6, 7, 8, 9^ Given their involvement in the initiation, progression, and metastasis of human cancers, some of these miRNAs have become studies of great interest. For example, it has been shown that levels of miR-143 and miR-145 tend to be lower in CRC tissue than in normal tissue.^10^ Moreover, it was also reported that miR-143 and miR-145 function as tumor suppressors through the repression of KRAS translation in human CRC.^10^ These findings suggest a close relationship between miRNAs and the development of CRC. Therefore, there is an urgent need to search for novel miRNAs aberrantly expressed and to investigate their complicated roles in CRC.

CRC is the second most common cause of cancer mortality worldwide and is the second and third most commonly diagnosed cancer in women and men, respectively.^11, 12^ Despite current therapy protocols that rely on surgical resection, pre- and postoperative chemotherapy and molecular-targeting therapy agents, tumor reccurrence and liver metastasis are common in patients with CRC, which essentially dictates the survival of patients with CRC.^13^ Hence, to identify new therapeutic targets is imperative for the improvement of therapeutic approaches for patients with CRC.

The nuclear factor 90 (NF90) family is known to be transcribed from the interleukin enhancer-binding factor 3 (ILF3) gene.^14^ The two most prominent protein isoforms are termed NF90 (also known as DRBP76 and NFAR1) and NF110 (also known as ILF3, NFAR2, and TCP110), and have apparent molecular masses of 90 and 110 kDa, respectively.^14^ Although both NF90 and NF110 are homologous in the N-terminal and central regions, their C-terminal are completely different.^14^ NF90 was originally purified as a DNA-binding complex regulating the interleukin-2 (IL-2) promoter.^15^ However, its function is not restricted to T cells because NF90 was found to regulate a number of other mRNAs. In addition, it is involved in regulating protein translation, DNA repair, RNA processing, host resistance to viral infections, and mitosis.^16^ Recently, NF90 was found to affect breast cancer angiogenesis and NF90/NF45 complex also mediates E6 oncogene expression in human papilloma virus-transformed cervical carcinoma cells.^17^ However, little is known about its role and regulation in CRC.

Altered expression of microRNA-590-5p (miR-590-5p) is involved in tumorigenesis, and it has been reported that miR-590-5p may function as oncogenes or tumor suppressors in cervical cancer and renal carcinoma, respectively.^18, 19^ However, its role in CRC remains to be determined. In this study, we sought to determine whether miR-590-5p can regulate angiogenesis, growth and metastasis of CRC, and its target gene.

## Results

### miR-590-5p expression in human CRC is decreased and is significantly correlated with poor survival

To determine the potential functions of miR-590-5p in CRC pathogenesis, we analyzed miR-590-5p expression in normal human intestinal epithelial cells (HIECs) and several CRC cell lines, which included the following: SW620, HCT116, HT29, SW480, and LOVO. Expression of miR-590-5p was lower in CRC cells than normal HIECs (Figure 1a). Consistently, miR-590-5p expression was significantly decreased in CRC tissues compared with normal colorectal tissues (Figure 1b). To investigate the clinical significance of miR-590-5p downregulation in CRC, we further analyzed the relationship between clinicopathologic features and miR-590-5p expression levels in CRC cases. Importantly, we found that downregulation of miR-590-5p expression was associated with larger tumor size or lymph node metastasis (Table 1). In addition, it was observed that miR-590-5p expression was significantly correlated with CRC severity (Figure 1c). Clinically, Kaplan–Meier test indicated that patients with low miR-590-5p expression exhibited significantly shorter survival time (Figure 1d). Altogether, these findings demonstrate a close association between miR-590-5p downregulation and poor CRC prognosis, and suggest that miR-590-5p may function as a tumor suppressor in CRC development.

### miR-590-5p inhibits CRC angiogenesis

Given that angiogenesis is an integral component of aggressive CRC, we explored whether miR-590-5p has a role in CRC angiogenesis. After immunohistochemical analysis, we observed significantly higher levels of CD31 (a marker for microvessels denoting enhanced angiogenesis) tumors from the SW480-miR-590-5p inhibitor group than tumors from the control scramble group (Figure 2a). We found a significant downregulation in CD31 expression in tumors from the SW620-miR-590-5p group compared with that from the SW620-control (Figure 2a), suggesting miR-590-5p may have antiangiogenic properties in CRC. In addition, tumor volume from the SW480-miR-590-5p inhibitor and SW620-scramble groups was significantly higher than those from SW480-scramble and SW620-miR-590-5p groups, respectively (Figure 2b). We utilized the chick embryo chorioallantoic membrane (CAM) assay to further characterize the effect of miR-590-5p on CRC angiogenesis and found that the SW480-scramble and SW620-miR-590-5p groups, had significant new blood vessel formation when compared with the SW480-miR-590-5p inhibitor and SW620-scramble (Figures 2c and d). The effect of miR-590-5p on CRC angiogenesis was further confirmed by *in vitro* endothelial cell tube formation assays. As compared with the conditioned media (CM) from the SW480-scramble and SW620-miR-590-5p clones, CM from the SW480-miR-590-5p inhibitor and SW620-Scramble groups significantly promoted tube formation (Figures 2e and f). Together, our data indicate that miR-590-5p is a potent inhibitor of CRC angiogenesis.

### miR-590-5p reduces angiogenesis by downregulating vascular endothelial growth factor (VEGFA)

To identify the angiogenic factors regulated by miR-590-5p, we used an antibody array in which levels of secreted angiogenic factors were compared in the CM of CRC cells with and without overexpression of miR-590-5p. This array highlighted a twofold differential in VEGFA production (Figure 3a). Although VEGFA has at least nine subtypes (VEGFA_121_, VEGFA_145_, VEGFA_148_, VEGFA_162_, VEGFA_165_, VEGFA_165_b, VEGFA_183_, VEGFA_189_, and VEGFA_206_) owing to the alternative splicing of a single gene, we only focused on VEGFA_165_ isoform because it has a central role in vascular development.^20^ The induction of VEGFA was further confirmed and quantified by enzyme-linked immunosorbent assay (ELISA) studies on miR-590-5p-deleted cells grown in CM. The VEGFA level was significantly higher in the miR-590-5p inhibitor SW480 cells when compared with the control cells, whereas miR-590-5p overexpression reduced VEGFA level in SW620 cells (Figure 3b). Given that VEGFA showed a robust change, we further investigated the role of VEGF in miR-590-5p knockdown-induced angiogenesis. SW480 and HT29 miR-590-5p-deficient cells were transfected with either scramble or VEGFA siRNA, and the CM was evaluated in CAM and HUVEC differentiation assays. Compared with the control, scrambled siRNA, VEGFA siRNA markedly inhibited neovascularization in CAM and HUVEC tube formation by the CM from miR-590-5p-deleted CRC cells (Figures 3c and d), thus supporting our suggestion that the high levels of angiogenesis induced by miR-590-5p knockdown were dependent on the elevated VEGFA levels.

### miR-590-5p inhibits CRC tumor angiogenesis by directly targeting NF90

VEGFA does not contain a miR-590-5p target sequence and is unlikely to be a direct target of miR-590-5p. To delineate the mechanisms driving CRC aggressive behavior once miR-590-5p was inhibited, we employed several bioinformatics tools such as TargetScan, miRanda, and PicTar were used to identify potential target genes. We focused on NF90 because it is an angiogenesis-related gene and there exists a highly conserved miR-590-5p-targeting sequence within 3'-UTR of NF90 (Figure 4a). NF90 was known to enhance VEGFA expression, thereby promoting cancer growth and metastasis.^21^ To demonstrate if NF90 was a direct target of miR-590-5p in CRC cells, we conducted luciferase reporter assays after transfection of wild-type (wt) and mutated NF90 3′-UTR into CRC cells with synthetic miR-590-5p mimic. As shown in Figure 4a, overexpression of miR-590-5p significantly reduced the expression of a luciferase reporter fused to wild-type NF90 miR-590-5p-targeting sequence, but did not affect the expression of a reporter with mutated sequence. Upon overexpressing miR-590-5p, the levels of NF90 mRNA and protein were substantially decreased in SW620 cells but miR-590-5p sponge inhibitor was able to increase the NF90 protein and mRNA levels (Figures 4b and c).

In order to understand if miR-590-5p-dependent suppression of NF90 was mediated by a miRNA-dependent pathway, we compared the expression of NF90 in wild-type HCT116 cells and Dicer, a miRNA biogenesis essential protein, deficient HCT116 cells. As expected, overexpression of pre-miR-590 was able to reduce NF90 expression in wild-type cells, but not in HCT116 Dicer-deficient cells (Figure 4d), suggesting that NF90 downregulation is primarily owing to miR-590-5p-dependent post-transcriptional repression. These results indicate that NF90 is a direct target of miR-590-5p in CRC.

To demonstrate that miR-590-5p/NF90 axis affects CRC angiogenesis via regulating VEGFA expression, we increased and decreased miR-590-5p and NF90 expression, respectively. It was observed that enhanced expression of NF90 in SW480 cells promoted HUVECs migration, invasion, and proliferation (Supplementary Figure 1A-D), whereas knockdown of endogenous NF90 in SW620 inhibited these behaviors (Supplementary Figure 1E-H). In SW620 cells, we found that ectopic expression of NF90 significantly counteracted the inhibition of HUVEC migration, invasion, and proliferation caused by overexpression of miR-590-5p. In SW480 cells, we observed a similar phenomenon, which could be reversed by reducing NF90. Furthermore, similar trends were observed in tube formation and CAM assay (Supplementary Figure 2) and when we checked the levels of VEGFA and NF90 protein (Figures 4e and f). We also investigated the other members of VEGF family: VEGF-B, VEGF-C,VEGF-D, and VEGF-E using their specific antibodies. As shown in Figure 4e (right panel), NF90 does not affect their expression levels. These results confirmed our hypothesis that miR-590-5p in CRC cells reduces angiogenesis and VEGF expression by inhibiting NF90 expression.

To investigate whether reduced miR-590-5p expression clinically correlates with increased levels of NF90 in CRC tissues, 20 pairs of primary CRC samples were compared with adjacent normal tissues to determine NF90 protein levels using western blotting analysis. The results showed that levels of NF90 protein in CRC samples were dramatically higher than in adjacent normal tissues (Figure 4g). Moreover, linear correlation analysis showed an inverse correlation between miR-590-5p and NF90 expression in CRC tissues, indicating that decreased expression of miR-590-5p was significantly correlated with increased NF90 protein expression in this set of CRC tissues (Figure 4h).

### Inhibition of NF90 profoundly abrogates tumorigenesis and metastasis of CRC Cells *in vivo*

Next, we investigated the impact of NF90 on CRC carcinogenesis *in vivo*. SW620 cells stably transfected with shNF90 or vector alone (shcontrol) were subcutaneously injected in 5-week-old severe combined immunodeficient (SCID) mice and the tumor growth over 4 weeks was monitored. Quantitative RT-PCR and immunoblot indicated downregulated NF90 expression in shNF90 stably transfected cells (Figure 5a). Knockdown of NF90 significantly decreased the potential of SW620 cells to develop tumors *in vivo* (Figure 5b). Moreover, relative to control cells, deletion of NF90 significantly reduced tumor volume (Figure 5c) and tumor weight in NF90 knockdown cells (Figure 5d). For *in vivo* imaging analysis, luciferase transfected control and shNF90 cells were subcutaneously injected into mice. We observed increased tumor growth 3 weeks after injection with control SW620 cells and significant tumor regression in mice injected with shNF90 cells (Figure 5e), thus suggesting that NF90 knockdown rescues the tumorigenic potential of aggressive CRC cells.

The impact of NF90 expression on the metastasis potential of CRC cells *in vivo* was monitored. As shown in Figure 5f, compared with those in the control group, mice injected with shNF90 had fewer lung metastases (left panel). The histological photomicrographs of lung tissue sections from each mouse were H&E stained, which further confirms lung metastases (right panel). In summation, these results indicated that NF90 was sufficient to promote lung metastasis of CRC.

### Knockdown of NF90 leads to a reduction of pri-miR-590 and an increase of mature miR-590-5p

NF90 was shown to function as a negative regulator in miRNA biogenesis.^22^ When NF90 was overexpressed, primary miRNA (pri-miRNA) processing into precursor miRNA (pre-miRNA) was inhibited.^22^ Therefore, we questioned whether NF90 could affect the expression levels of miR-590-5p in CRC. We then measured the levels of pri-miR-590 and mature miR-590-5p, which were produced from tested pri-miR-590 in NF90 knockdown cells. Transfection of siRNAs targeting NF90 caused ~85% inhibition of the expression of endogenous NF90 protein (Figure 6a). As expected, a significant decrease in pri-miR-590 in the NF90 knockdown cells was observed (Figure 6b), whereas mature miR-590-5p was increased in cells that were depleted of NF90, in accordance with the decrease in pri-miR-590 (Figure 6c). Overexpression of NF90 increased pri-miR-590 and decreased mature miR-590-5p in CRC cells (Figures 6d–f). As the NF90-NF45 complex impairs pri-miRNA processing and binds to pri-miRNA,^22^ we hypothesized that the binding of NF90 to pri-miR-590 reduces the accessibility of Drosha-DGCR8 to pri-miR-590, resulting in the inhibition of pri-miR-590 processing. To test this idea, we performed an electrophoretic mobility shift assay (EMSA) using recombinant NF90 and pri-miR-590 probe. As expected, the EMSA probed with pri-miR-590 clearly showed that NF90 bound to it *in vitro* compared with the control (Figure 6g), implying that overexpressed NF90 has the ability to associate with endogenous pri-miR-590. Together, these results suggest a negative feedback loop between NF90 and miR-590-5p (Figure 6h) and confirm that NF90 negatively regulates the level of miR-590-5p in CRC.

## Discussion

For the following reasons we focused our attention mainly on the function of miR-590-5p. First, we found that the expression of miR-590-5p was significantly lower in the human CRC cells and tissues than in the normal controls. Second, miR-590-5p is a novel miR, and very little was known about its function. Thirdly, it has been reported that miR-590-5p may function as oncogenes or tumor suppressors in cervical cancer and renal, respectively,^18, 19^ however, very little was known about its role in CRC. The current study demonstrated a critical role for miR-590-5p in CRC angiogenesis and development. The level of miR-590-5p expression was found to be significantly lower in CRC tissue than that in normal colon tissue, and miR-590-5p expression was lower in metastatic compared with non-metastatic CRC. We also demonstrated that miR-590-5p inhibited CRC cell proliferation, migration, and angiogenesis by suppressing NF90-VEGF axis. It is clear that NF90 can inhibit the levels of mature miR-590-5p and completely reversed the effects of miR-590-5p on CRC suppression, suggesting a negative feedback loop between NF90 and miR-590-5p. These phenomena were further validated in a mice tumor xenograft model. Our results offered new insights into the regulation of CRC, challenging previous studies that reported two opposite roles of miR-590-5p in tumorigenesis. On the one hand, miR-590-5p was downregulated in breast cancer samples and could inhibit its metastasis,^23^ it was found that miR-590-5p levels in hepatocellular carcinoma (HCC) patients were inversely associated with tumor size, stage, epithelial–mesenchymal transition (EMT), and metastasis by targeting S100A1,^24^ which suggests its negative role in tumor development. However, miR-590-5p was found to be upregulated in the examined renal cell carcinoma cell lines and seem to function as an oncomir by targeting PBRM1,^18^ whereas miR-590-5p acts as an oncogene by targeting the CHL1 gene and promotes cervical cancer proliferation.^19^ In the current study, we found that compared with non-metastatic and normal samples, miR-590-5p expression was downregulated in CRC specimens and CRC cell lines. Functional assays demonstrated that miR-590-5p inhibited CRC proliferation and lung metastasis. For the first time, we found that miR-590-5p and its new target NF90 directly established a negative feedback loop to affect CRC angiogenesis via VEGF. Our results suggest, miR-590-5p suppressed CRC metastasis by inhibiting NF90/VEGF, which is also a contributor to EMT. However, further studies are needed to determine if EMT-related proteins are regulated by miR-590-5p.

Accumulating evidence established that miRNAs functions as effective molecular biomarkers for cancer diagnosis, prognosis, and therapy.^25^ miRNA-CHIP assays has indicated that many miRNAs were aberrantly expressed in CRC.^26^ Several steps were involved in the biogenesis of miRNAs.^27^ First, pri-miRNAs are transcribed from miRNA genes by RNA polymerase II. Then a microprocessor complex composed of Drosha and DGCR8 processes pri-miRNAs into pre-miRNAs. Subsequently, the pre-miRNAs are exported to the cytoplasm and cleaved into mature miRNA duplexes by the Dicer complex. Thereafter, mature miRNA is loaded into the RNA-induced silencing complex, binds to target mRNAs and results in their translational suppression or protein degradation. Recently, several oncogenes were identified as new regulators of the biogenesis of miRNAs. For example, it was reported that some RNA-binding proteins (Lin28A/B, the Musashi homolog 2/Hu antigen R complex) negatively regulated miRNA biogenesis.^28, 29^ They inhibited miRNA processing by associating with pri- or pre-miRNAs. The inhibition of the miRNA processing pathway was recently demonstrated to lead to various human diseases. Lin28A/B enhances the growth of breast and colon tumors via inhibition of let-7 miRNA biogenesis.^30^ These reports strongly support our current data: we indicated that NF90 induces CRC angiogenesis, growth, and metastasis through suppression of pri-miR-590 processing by binding of NF90 to pri-miR-590, thus decreasing the levels of mature miR-590-5p. Interestingly, it has been reported that NF90 or the NF90-NF45 complex is involved in mRNA stabilization and transcription. Consistent with previous reports that NF90 functions as an AU-binding protein to regulate IL-2, VEGF, or cyclin E1,^31, 32^ our results suggested that NF90 indeed regulates VEGF in CRC tissues in the similar manner. We showed that altering NF90 levels had a clear effect on the half-life of VEGF mRNA. Moreover, the level of NF90 has been reported to be elevated in non-small-cell lung, epithelial ovarian, and breast cancers.^17, 33^ Here, we also observed a significant increase of NF90 expression level in CRC compared with that in adjacent normal tissues. Given that NF90 has a role in the promotion of tumorigenesis, it is possible to suggest that once upregulated by miR-590-5p knockdown, the NF90-mediated feedback loop will allow CRC cells to become more autonomous. This would enhance the ability of CRC cells to proliferate, invade, and metastasis to new microenvironments, which may explain the strong pro-metastasis phenotype we have observed. Noteably, although NF90 protein functions as a negative regulator in miRNA biogenesis, so far there is no reports about others miR which could regulate NF90. But there are several miRNAs,^34, 35, 36^ which could regulate VEGF and they express/modulate in CRC.

In summary, we demonstrated that miR-590-5p was downregulated in CRC tissues compared with normal tissues, and especially in metastatic compared with non-metastatic CRC. miR-590-5p impaired cell proliferation, migration, and tumor angiogenesis mainly by inhibiting NF90/VEGFA axis *in vitro* and *in vivo*. The results of this study greatly improve our understanding of the regulation of CRC development and provide potential new therapeutic targets for the management of CRC.

## Materials and Methods

### Cell culture and transfection

The normal HIEC line, CRC cell lines (HT29, LOVO, SW620, and SW480) and human embryonic kidney (HEK) 293 T cell line were purchased from the Type Culture Collection of the Chinese Academy of Sciences (Shanghai, China), and HCT116 cell line was purchased from Shanghai Institute of Biochemistry and Cell Biology (China). All the cell lines were cultured in Dulbecco's modified Eagle's medium (DMEM; Hyaline, UT, USA) with 10% fetal bovine serum (Gibco, Carlsbad, CA, USA) at 37 °C in an incubator supplemented with 5% CO_2_.

The *Homo sapiens* miR-590-5p mimic, miR-590-5p inhibitor, mimic negative control, and inhibitor negative control (scramble) sequences and human NF90 and VEGFA small-interfering RNA (siRNA) were from GenePharma (Shanghai, China). The NF90 expression plasmid (pCMV-EGFP-NF90) was from GeneChem (Shanghai, China). Indicated cells were transfected using Lipofectamine 2000 (Invitrogen) according to the manufacturer's instructions. For stable expression of miR-590-5p, indicated cells were transfected with the miR-590-5p expression plasmid (pCMV-pre-miR-590, Origene) using Lipofectamine 2000 (Invitrogen) and selected with 1 mg/ml G418 (Sigma). For stably knockdown NF90, cells were infected with phU6-puro-NF90-shRNA lentivirus particles (GeneChem) and selected with 1 mg/ml puromycin (Sigma).

### RNA isolation and quantitative real-time PCR analysis

To detect miR-590-5p expression in CRC, the MicroRNA TaqMan Reverse Transcription Kit and the TaqMan MicroRNA Assays (Applied BioSystems, USA) was used. The relative expression level of miR-590-5p was determined by quantitative RT-PCR using mirVana qRT-PCR microRNA Detection Kit (Genecopoeia, China) as described in the manufacturer's instructions. The expression of each target gene was normalized to that of U6 snRNA. The following primers were used for quantification of human U6 snRNA and has-miR-590-5p respectively: U6 snRNA: 5′-GTGCTCGCTTCGGCAGCACAT-3′ and 5′-TACCTTGCGAAGTGCTTAAAC-3′ and hsa-miR-590-5p: 5′-GAGCTTATTCATAAAAGT-3′ and 5′-TCCACGACACGCACTGGATACGAC-3′. Total RNA was extracted using Trizol reagent (Invitrogen). Reverse transcription was performed using the First Strand cDNA Synthesis Kit (Takara, Japan). Quantitative PCR (qPCR) was performed using an ABI Prism 7900HT Sequence Detection System (Applied Biosystems) with SYBR Premix Ex Taq II (Takara). Quantification was calculated using the 2−ΔΔCT method and is presented as fold change. Primer sequences were as follows: NF90: (forward), 5′GATGGCAATTCATTCGAGGC3′, (reverse), 5′GCAAGAGCAGCGTAGGCCTTC3′ GAPDH: (forward), 5′CTGGTAAAGTGGATATTGTTG3′, (reverse), 5′GAGGCTGTTGTCATACTTCTC3′.

### MiR-590-5p *in situ* hybridization

In all, 6 *μ*m-thick paraffin sections were mounted on Superfrost glass slides, de-paraffinized, treated with 15 *μ*g/ml proteinase-K for 7.5 min at 37 °C, then immersed into 3% hydrogen peroxide/phosphate buffered saline for peroxidase blocking for 15 min and dehydrated in new ethanol solutions. One hundred microliter hybridization mix 50 nM double-DIG LNA miR-590-5p probe (positive control test: 1 nM LNA *U6* snRNA probe; negative control test: 50 nM Scramble probe) (Invitrogen) was applied onto the slides. The slides were incubated overnight at 56 °C, then washed twice with 5 × SSC buffer for 5 min at RT and treated by 5 min stringent wash steps at 56 °C in 1 × SSC buffer twice followed by 0.2 × SSC buffer once. Then, the slides were immersed into 0.2 × SSC buffer for 5 min at RT, and incubated with blocking solution (Roche, Germany) with 2% sheep serum at RT for 15 min. Sheep anti-DIG-horseradish peroxidase (HRP) conjugate (BIO-RAD) was applied diluted at 1:50 for 15 min at RT. Digoxogenin-labeled tyramide was then applied at 1:50 dilution for 30 min at RT, followed by the incubation with sheep anti-DIG-HRP conjugate at 1:100 for 30 min at RT. The hybridization signal was confirmed using the HRP substrate 3-amino-9-ethylcarbazole (Dako, USA) for 5 min and counterstained with hematoxylin for 5 min at RT. Finally, the slides were mounted directly with 1–2 drops of aqua mount (Dako) and air-dried. The images were photographed at 200 × with microscope (Olympus). The staining intensity was evaluated according to an established criteria^37^ and normalized with U6 signals.

### Western blotting

Indicated cells were lysed in Radio-Immunoprecipitation Assay buffer (Pierce, Rockford, IL, USA), and protein concentrations in the lysates were determined by the BCA method. Forty micrograms of total protein were separated on 10% SDS–PAGE gels and transferred to PVDF membranes (Fisher, Waltham, MA, USA). After blocking with 5% milk powder diluted in TBS containing 0.05% Tween 20 (TBST), membranes were probed with indicated primary antibodies (NF90, Abcam, Cambridge, MA, USA, ab92355; VEGFA, Abcam-ab46154, VEGF-B, Santa Cruz, Dallas, TX, USA, sc13083; VEGF-C, Santa Cruz-sc9047; VEGF-D, Santa Cruz-sc13085; VEGF-E, Santa Cruz-sc18228, and *α*-Tubulin, Sigma-T6199). HRP-conjugated secondary antibody (BIO-RAD) and an enhanced chemiluminescence system (Pierce) were used for detection.

### CAM assay

In brief, fertilized chicken eggs were kept in a humidified incubator at 37 °C for 3 days. Approximately 4–5 ml egg albumin was removed with a hypodermic needle. A 2.5-cm diameter window was made with a razor and a 1% solution of methylcellulose containing various tumor cell CM was loaded inside a silicon ring that was placed onto the surface of CAM. Two days later, 2–3 ml intralipose was injected beneath the CAM, and the membrane was observed at 10 × under a microscope and the total number of vessel branch points directly beneath the disc was counted.

### HUVEC tube formation assay

HUVECs from American Type Culture Collection were cultured in endothelial cell growth medium (Invitrogen). One hundred microliter of undiluted matrigel was layered in a 96-well plate for 3 h. Then HUVEC cells (1 × 10^5^ cells/ml) were trypsinized, washed with PBS, and added to the precoated 96-well plates together with the indicated CM treatment. Eighteen hours later, the tubes were observed and photographed at 100 × under Nikon Eclipse TE2000E inverted microscope (Nikon, Tokyo, Japan). The Number of vessel branch points of tube per field was counted from the digital images. Results are expressed as means±S.D.

### Migration assay

HUVEC cells (5 × 10^4^ cells/filter) were plated on a polycarbonate filter of 8 *μ*m-pore size of the transwell insert and incubated at 37 °C for indicated time, and cells were visualized by crystal violet staining. The uncoated upper side of each filter was wiped with a cotton swab to remove cells that had not migrated through the filter. Migrated cells were counted. Results are expressed as means±S.D.

### Luciferase reporter assay

A fragment of 3′-UTR of NF90 containing the putative miR-590-5p-binding site was amplified by PCR and inserted at the *Xol* I and *Not*I restriction sites, immediately downstream of the luciferase gene in the psiCHECK-2 vector (Promega, Madison, WI, USA). The primers were used as followed: wt-NF90 (forward) 5′-CCGGCTCGAGATCTCCCACATTCATACC-3′, (reverse) 5′-TAAGCGGCCGCTTCATTAGCAGAAACCC-3′. A 3′-UTR of NF90 construct with a mutant seed sequence of miR-590-5p was also generated using the primers: mut-NF90 (forward) 5′-GTCAAAGGGGCCTGAGAAAAGAATG-3′, (reverse) 5′-TAAGTTGCACCTCAGAGTGCAAACA-3′. All constructs were verified by DNA sequencing. HEK-293 T cells and CRC cells were seeded in 48-well plates (2 × 10^3^ per well). After 24 h incubation, Lipofectamine 2000 (Invitrogen) were used to transfected indicated cells with 100 nM psiCHECK-2-NF90 3′UTR or psiCHECK-2-mut-NF90 3′UTR with control oligonucleotide or mimic according to the manufacturer's protocol. Forty-eight hours later, the Dual Luciferase Reporter Assay System (Promega) Luciferase activity was used to measure Firefly luciferase activity. All experiments were performed in triplicate and repeated three times independently.

### ELISA

An ELISA based angiogenesis antibody array (Quantibody Human Angiogenesis Array 1, RayBiotech, Norcross, GA, USA) was used to determine the expression of angiogenic factors from CM secreted by SW620 cells transfected with miR-590-5p. The level of VEGF protein from indicated CM was determined with Human VEGFA_165_ ELISA Kit (RayBiotech) according to the manufacturer's instructions.

### EMSA

EMSA was performed as described previously.^22^ In brief, pri-miR-590 was amplified from 293 T cDNA by PCR with specific primers. The PCR products were subcloned into the pGEM-T-easy vector (Promega). The plasmids were linearized with SpeI and used for *in vitro* transcription to make ^32^P-radiolabeled RNA probes. Recombinant protein NF90 was preincubated with the labeled probe at 0 °C for 20 min and then electrophoresed on a 4% polyacrylamide gel containing 10% glycerol in 0.5 × Tris-borate-EDTA. Images were captured and intensities of specific bands were measured using a BAS-2500 imaging system (Fuji Film, Tokyo, Japan).

### Animal studies

All the animal experiments strictly adhered to the Regulations for the Administration of Affairs Concerning Experimental Animals, the Chinese national guideline for animal experiment. All procedures involving animals and their care in this study were approved and performed by the Harbin Medical University Institutional Animal Care and Use Committee. The cells were harvested by trypsinization, washed twice with cold serum-free medium, and re-suspended with 200 *μ*l serum-free medium. To evaluate cancer growth *in vivo*, 2 × 10^6^ indicated cells were independently injected subcutaneously into the back of SCID mice (Vital Rivers, Beijing, China) to establish tumor model. Then the mean tumor weight was measured and tumor volume was determined by the formula: tumor volume (mm^3^)=1/2 (*xy*^2^); *x* is the greatest longitudinal diameter and *y* is greatest transverse diameter. For *in vivo* imaging analysis, the control and shNF90 cells with stably expressing luciferase was subcutaneously injected in mice. Mice were injected i.p. with 150 mg/kg luciferin 15 min prior to imaging. Bioluminescence imaging was performed using the Xenogen IVIS Spectrum Imaging System (Caliper Life Sciences, Hopkinton, MA, USA). For detecting lung metastases, shNF90 SW620 cells and their control cells were injected by way of the tail vein into SCID mice (*n*=10 of each group). Lungs were collected and the surface nodules were counted. H&E was performed for histological examination. Data are expressed as mean ±S.D. The results are representative of three independent experiments.

### Clinical specimens

Primary CRC and corresponding normal tissue were collected and frozen in liquid nitrogen after resection between June 2008 and March 2010 in accordance with a protocol approved by the Ethical Committee of The First Affiliated Hospital of the Harbin Medical University. All patients provided written informed consent for the use of their tissues, according to the Declaration of Helsinki. The TNM stage of the tumor was determined according to the classification proposed by the AJCC Cancer Staging Manual. No patient in the current study received chemotherapy or radiation therapy before the surgery.

### Immunohistochemistry

The section was de-paraffinized and boiled in 10 mM citrate buffer (pH 6.0) for antigen retrieval. Endogenous peroxidase was blocked by 3% H_2_O_2_. Then slides were blocked in serum, incubated with the indicated antibodies at 4 °C overnight, then incubated with anti-rabbit secondary antibody, and visualized with diaminobenzadine (Sigma). Negative control was also performed. The images of IHC staining were photographed at 200 × with microscope (Olympus).

### Statistical analyses

Statistical analyses were performed using the SPSS statistical software 17.0 (SPSS Inc, Chicago, IL, USA). Normally distributed data are presented as mean±S.D. of at least three independent experiments. Statistical significance was evaluated by one-way analysis of variance with Student's *t*-test. Categorical variables were compared using *χ*^2^ or Fisher's exact test. Spearman correlation analysis was used for ranking correlation tests. The Kaplan–Meier and log-rank tests were used for the cumulative survival analysis. *P<0.05, **P<0.01, and ***P<0.0001.

## Figures and Tables

**Figure 1:** Downregulation of miR-590-5p in CRC and its association with poor survival. (**a**) Compared with the normal HIECs, quantitative RT-PCR was used to analyze relative expression of miR-590-5p in CRC cell lines. (**b**) Analysis of miR-590-5p *in situ* hybridization (ISH) signal in a group of 60 normal and paired CRC tissues (left panel). The level of miR-590-5p was estimated and compared between normal and cancer tissues (right panel). (**c**) Quantitative RT-PCR was used to measure the relative expression of miR-590-5p in the CRC tissues of different tumor TNM stages. (**d**) Kaplan–Meier survival test was used to detect the correlationship between the levels of miR-590-5p expression and survival of CRC patients. *P<0.05, **P<0.01, and ***P<0.0001

**Figure 2:** MiR-590-5p inhibits CRC angiogenesis. (**a**) *S*ubcutaneous CRC xenografts were established in nude mice using SW480-scramble, SW480-miR-590-5p inhibitor, SW620-control, or SW620-miR-590-5p cells, respectively. Then these tumor sections were stained with anti-CD31 (upper panel) and anti-DIG (lower panel) antibodies. (**b**) Graphical representation of tumor volume monitored after 4 weeks. (**c**) The indicated CM were loaded onto CAM, and the representative pictures were presented. (**d**) The new blood vessel formation in CAM was quantified. (**e**) The CM from the indicated cells were used to treat HUVECs, and tube formation was photographed, and (**f**) quantified. *P<0.05, **P<0.01

**Figure 3:** Increased VEGFA production contributes to enhanced angiogenesis of CRC induced by miR-590-5p knockdown. (**a)** Measurement of angiogenic factors secreted by CRC cells with overexpression of miR-590-5p. Serum-free CM from indicated cell monolayers was assayed by an angiogenesis antibody array, displaying differential in secreted VEGF. (**b**) ELISA was used to determine the VEGFA levels in the CM of the indicated cells. (**c** and **d**) Indicated cells depleted of miR-590-5p were transfected either with control siRNA or VEGFA siRNA, and the CM was subjected to CAM assay and tube formation assay. **P<0.01

**Figure 4:** MiR-590-5p inhibits VEGFA expression and CRC angiogenesis by repressing NF90. (**a**) Schematic representation of the putative miR-590-5p target site within the 3'-UTR of NF90 was shown on the top. Mutations used for abolishing miR-590-5p recognition sequence were highlighted in red. (Bottom) SW620 cells were transfected with control or pre-miR-590 plasmid along with WT or mutant NF90 luciferase reporter as shown. The activity of both Renilla and Firefly luciferases was assayed using the dual-luciferase reporter assay system. (**b** and **c**) Indicated cells were, respectively, transfected with pre-miR-590 or miR-590-5p inhibitor or their control plasmids. α-tubulin was used as loading control, and the levels of NF90 mRNA and protein expression were determined by qRT-PCR and western blot, respectively. (**d**) NF90 expression was determined by western blot in HCT116 Dicer+/+ and Dicer−/− cells transfected with control or pre-miR-590. (**e** and **f**) Western blotting assay was used to analyze the protein levels of VEGF and NF90 in indicated CRC cells. (**g**) NF90 expression was determined by western blot in CRC and adjacent tissues. (**h**) Linear correlation analysis was used to detect the correlationship between the levels of miR-590-5p and NF90 expression. *P<0.05, **P<0.01

**Figure 5:** NF90 knockdown reverses the tumorigenic growth *in vivo.* (**a**) Immunoblot (upper panel) and qRT-PCR (lower panel) showing expression of NF90 knockdown in CRC cells in comparison with control cells. (**b**) Five weeks old SCID mice were injected subcutaneously with SW620-control cells and shNF90 cells and tumors were monitored for 4 weeks. (**c**) Graphical representation of tumor volume monitored for 4 weeks. (**d**) Tumor weight in control and shNF90 mice. (**e**) *In vivo* imaging analysis indicates tumor burden in control mice compared with shNF90 mice. (**f**) *In vivo* animal model experiments were performed by injecting shNF90 SW620 cells into SCID mice via the tail vein to confirm the impact of NF90 on tumor metastasis. Representative gross and H&E-staining pictures (left panel) and the number of lung surface metastatic foci detected in each group (right panel, *n*=10/group). **P<0.01, ***P<0.0001

**Figure 6:** Knockdown of NF90 decreases pri-miR-590 and increases mature miR-590-5p. (**a**) whole-cell lysates were prepared from SW620 cells transfected with the indicated siRNAs and analyzed by immunoblotting with anti-NF90 and anti-α-tubulin antibodies. (**b**) The amount of pri-miR-590 was analyzed using qRT-PCR. GAPDH functioned as an internal control. (**c**) RNAs were isolated from SW620 cells transfected with the indicated siRNAs and analyzed for the amount of mature miR-590-5p. U6 was used as an internal control. (**d**) Whole-cell lysates were prepared from SW480 cells and analyzed by immunoblotting with anti-NF90 and anti-*α*-tubulin antibodies. (**e** and **f**) The amount of pri-miR-590 and mature miR-590-5p were analyzed by qRT-PCR. (**g**) NF90 binds to pri-miR-590 *in vitro*. EMSA was performed with the pri-miR-590 probe and without (−) or with recombinant NF90 protein alone at the indicated protein concentrations. *P<0.05, **P<0.01, and ***P<0.0001

**Table 1:** Relationship between miR-590-5p expression and clinicopathologic features of CRC patients (*n*=60)

**Variable**	**Relative miR-590-5p expression**		***P*-value**
	**Low (*n*=30)**	**High (*n*=30)**	
*Gender*			*NS*
Women	12	14	
man	18	16	
			
*Age*			*NS*
<60	13	15	
≥60	17	15	
			
*Primary tumor sites*			*NS*
Ascending colon	4	7	
Transverse colon	2	1	
Descending colon	4	3	
Sigmoid colon	8	9	
Rectum	12	10	
			
*Histological differentiation*			*NS*
Well	8	6	
Moderate	17	18	
Poor	5	6	
			
*Tumor size*			*<0.01*
<5 cm	3	25	
≥5 cm	27	5	
			
*Lymph node metastasis*			*<0.01*
Yes	26	9	
No	4	21	
			
*Distant metastasis*			*NS*
Yes	10	5	
No	20	25	
			
*Tumor stage*			*<0.01*
I–II	4	19	
III–IV	26	11	

Note: CRC patients were divided into miR-590-5p ‘High' group (relative fold change of ‘low' group) and ‘Low' group according to the staining by *in situ* hybridization. NS, not significant between any groups. Differences among variables were assessed by *χ*^2^ or Fisher's exact *χ*^2^-test

## Abbreviations

AUBP: AU-binding protein
CAM: chick embryo chorioallantoic membrane
CM: conditioned media
CRC: colorectal cancer
EMSA: electrophoretic mobility shift assay
EMT: epithelial–mesenchymal transition
HIECs: human intestinal epithelial cells
ILF3: interleukin enhancer-binding factor 3
miRNAs: MicroRNAs
NF90: nuclear factor 90
pre-miRNA: precursor miRNA
pri-miRNA: primary miRNA
RISC: RNA-induced silencing complex
SCID: severe combined immunodeficient mice
UTR: untranslated region
VEGFA: vescular endothelial growth factor A

## References

[bib1] Giacca M, Zacchigna S. Harnessing the microRNA pathway for cardiac regeneration. J Mol Cell Cardiol 2015; pii S0022-2828: 30070–30075.10.1016/j.yjmcc.2015.09.01726431632

[bib2] Simmer F, Venderbosch S, Dijkstra JR, Vink-Börger EM, Faber C, Mekenkamp LJ et al. MicroRNA-143 is a putative predictive factor for the response to fluoropyrimidine-based chemotherapy in patients with metastatic colorectal cancer. Oncotarget 2015; 6: 22996–23007.2639238910.18632/oncotarget.4035PMC4673216

[bib3] Das AV, Pillai RM. Implications of miR cluster 143/145 as universal anti-oncomiRs and their dysregulation during tumorigenesis. Cancer Cell Int 2015; 15: 92.2642511410.1186/s12935-015-0247-4PMC4588501

[bib4] Pradhan M, Nagulapalli K, Ledford L, Pandit Y, Palakal M. A system biology approach for understanding the miRNA regulatory network in colon rectal cancer. Int J Data Min Bioinform 2015; 11: 1–30.2625537410.1504/ijdmb.2015.066332

[bib5] Tanaka S, Hosokawa M, Ueda K, Iwakawa S. Effects of decitabine on invasion and exosomal expression of miR-200c and miR-141 in oxaliplatin-resistant colorectal cancer cells. Biol Pharm Bull 2015; 38: 1272–1279.2617933310.1248/bpb.b15-00129

[bib6] Yang Y, Gu X, Zhou M, Xiang J, Chen Z. Serum microRNAs: a new diagnostic method for colorectal cancer. Biomed Rep 2013; 1: 495–498.2464897410.3892/br.2013.109PMC3917018

[bib7] Phua LC, Chue XP, Koh PK, Cheah PY, Chan EC, Ho HK. Global fecal microRNA profiling in the identification of biomarkers for colorectal cancer screening among Asians. Oncol Rep 2014; 32: 97–104.2484183010.3892/or.2014.3193

[bib8] Ogata-Kawata H, Izumiya M, Kurioka D, Honma Y, Yamada Y, Furuta K et al. Circulating exosomal microRNAs as biomarkers of colon cancer. PLoS One 2014; 9: e92921.2470524910.1371/journal.pone.0092921PMC3976275

[bib9] Chang KH, Mestdagh P, Vandesompele J, Kerin MJ, Miller N. MicroRNA expression profiling to identify and validate reference genes for relative quantification in colorectal cancer. BMC Cancer 2010; 10: 173.2042993710.1186/1471-2407-10-173PMC2873395

[bib10] Pagliuca A, Valvo C, Fabrizi E, di Martino S, Biffoni M, Runci D et al. Analysis of the combined action of miR-143 and miR-145 on oncogenic pathways in colorectal cancer cells reveals a coordinate program of gene repression. Oncogene 2013; 32: 4806–4813.2312839410.1038/onc.2012.495

[bib11] Haggar FA, Boushey RP. Colorectal cancer epidemiology: incidence, mortality, survival, and risk factors. Clin Colon Rectal Surg 2009; 22: 191–197.2103780910.1055/s-0029-1242458PMC2796096

[bib12] Herszényi L, Tulassay Z. Epidemiology of gastrointestinal and liver tumors. Eur Rev Med Pharmacol 2010; 14: 249–258.20496531

[bib13] Akgül Ö, Çetinkaya E, Ersöz S, Tez M. Role of surgery in colorectal cancer liver metastases. World J Gastroenterol 2014; 20: 6113–6122.2487673310.3748/wjg.v20.i20.6113PMC4033450

[bib14] Wandrey F, Montellese C, Koos K, Badertscher L, Bammert L, Cook AG et al. The NF45/NF90 heterodimer contributes to the biogenesis of 60 S ribosomal subunits and influences nucleolar morphology. Mol Cell Biol 2015; 35: 3491–3503.2624028010.1128/MCB.00306-15PMC4573712

[bib15] Shim J, Lim H, R Yates J, Karin M. Nuclear export of NF90 is required for interleukin-2 mRNA stabilization. Mol Cell 2002; 10: 1331–1344.1250400910.1016/s1097-2765(02)00730-x

[bib16] Patiño C, Haenni AL, Urcuqui-Inchima S. NF90 isoforms, a new family of cellular proteins involved in viral replication? Biochimie 2015; 108: 20–24.2544714410.1016/j.biochi.2014.10.022

[bib17] Shamanna RA, Hoque M, Pe'ery T, Mathews MB. Induction of p53, p21 and apoptosis by silencing the NF90/NF45 complex in human papilloma virus-transformed cervical carcinoma cells. Oncogene 2013; 32: 5176–5185.2320850010.1038/onc.2012.533PMC4032571

[bib18] Xiao X, Tang C, Xiao S, Fu C, Yu P. Enhancement of proliferation and invasion by MicroRNA-590-5p via targeting PBRM1 in clear cell renal carcinoma cells. Oncol Res 2013; 20: 537–544.2406328410.3727/096504013X13775486749335

[bib19] Chu Y, Ouyang Y, Wang F, Zheng A, Bai L, Han L et al. MicroRNA-590 promotes cervical cancer cell growth and invasion by targeting CHL1. J Cell Biochem 2014; 115: 847–853.2428817910.1002/jcb.24726

[bib20] Takahashi H, Shibuya M. The vascular endothelial growth factor (VEGF)/VEGF receptor system and its role under physiological and pathological conditions. Clin Sci 2005; 109: 227–241.1610484310.1042/CS20040370

[bib21] Vumbaca F, Phoenix KN, Rodriguez-Pinto D, Han DK, Claffey KP. Double-stranded RNA-binding protein regulates vascular endothelial growth factor mRNA stability, translation, and breast cancer angiogenesis. Mol Cell Biol 2008; 28: 772–783.1803985010.1128/MCB.02078-06PMC2223436

[bib22] Sakamoto S, Aoki K, Higuchi T, Todaka H, Morisawa K, Tamaki N et al. The NF90-NF45 complex functions as a negative regulator in the microRNA processing pathway. Mol Cell Biol 2009; 29: 3754–3769.1939857810.1128/MCB.01836-08PMC2698745

[bib23] Murria R, Palanca S, de Juan I, Alenda C, Egoavil C, Seguí FJ et al. Immunohistochemical, genetic and epigenetic profiles of hereditary and triple negative breast cancers. Relevance in personalized medicine. Am J Cancer Res 2015; 5: 2330–2343.26328265PMC4548346

[bib24] Shan X, Miao Y, Fan R, Qian H, Chen P, Liu H et al. MiR-590-5 P inhibits growth of HepG2 cells via decrease of S100A10 expression and Inhibition of the Wnt pathway. Int J Mol Sci 2013; 14: 8556–8569.2359841710.3390/ijms14048556PMC3645761

[bib25] Nair J, Jain P, Chandola U, Palve V, Vardhan NR, Reddy RB et al. Gene and miRNA expression changes in squamous cell carcinoma of larynx and hypopharynx. Genes Cancer 2015; 6: 328–340.2641321610.18632/genesandcancer.69PMC4575920

[bib26] Bullock MD, Pickard K, Mitter R, Sayan AE, Primrose JN, Ivan C et al. Stratifying risk of recurrence in stage II colorectal cancer using deregulated stromal and epithelial microRNAs. Oncotarget 2015; 6: 7262–7279.2578826110.18632/oncotarget.3225PMC4466683

[bib27] Orellana EA, Kasinski AL. MicroRNAs in cancer: a historical perspective on the path from discovery to therapy. Cancers 2015; 7: 1388–1405.2622600210.3390/cancers7030842PMC4586775

[bib28] Faria AM, Sbiera S, Ribeiro TC, Soares IC, Mariani BM, Freire DS et al. Expression of LIN28 and its regulatory microRNAs in adult adrenocortical cancer. Clin Endocrinol 2015; 82: 481–488.10.1111/cen.1260725200669

[bib29] Choudhury NR, de Lima Alves F, de,rés-Aguayo L, Graf T, Cáceres JF, Rappsilber J et al. Tissue-specific control of brain-enriched miR-7 biogenesis. Genes Dev 2013; 27: 24–38.2330786610.1101/gad.199190.112PMC3553281

[bib30] Suzuki HI, Katsura A, Miyazono K. A role of uridylation pathway for blockade of let-7 microRNA biogenesis by Lin28B. Cancer Sci 2015; 106: 1174–1181.2608092810.1111/cas.12721PMC4582986

[bib31] Reichman TW, Muñiz LC, Mathews MB. The RNA binding protein nuclear factor 90 functions as both a positive and negative regulator of gene expression in mammalian cells. Mol Cell Biol 2002; 22: 343–356.1173974610.1128/MCB.22.1.343-356.2002PMC134226

[bib32] Jiang W, Huang H, Ding L, Zhu P, Saiyin H, Ji G et al. Regulation of cell cycle of hepatocellular carcinoma by NF90 through modulation of cyclin E1 mRNA stability. Oncogene 2015; 34: 4460–4470.2539969610.1038/onc.2014.373PMC4433881

[bib33] Guo NL, Wan YW, Tosun K, Lin H, Msiska Z, Flynn DC et al. Confirmation of gene expression-based prediction of survival in non-small cell lung cancer. Clin Cancer Res 2008; 14: 8213–8220.1908803810.1158/1078-0432.CCR-08-0095PMC2605664

[bib34] Zhang D, Zhou J, Dong M. Dysregulation of microRNA-34a expression in colorectal cancer inhibits the phosphorylation of FAK via VEGF. Dig Dis Sci 2014; 59: 958–967.2437078410.1007/s10620-013-2983-4

[bib35] Qiu Y, Yu H, Shi X, Xu K, Tang Q, Liang B et al. MicroRNA-497 inhibits invasion and metastasis of colorectal cancer cells by targeting vascular endothelial growth factor-A. Cell Prolif 2016; 49: 69–78.2684037210.1111/cpr.12237PMC6495881

[bib36] Zhang W, Zou C, Pan L, Xu Y, Qi W, Ma G et al. MicroRNA-140-5p inhibits the progression of colorectal cancer by targeting VEGFA. Cell Physiol Biochem 2015; 37: 1123–1133.2640243010.1159/000430237

[bib37] Adams EJ, Green JA, Clark AH, Youngson JH. Comparison of different scoring systems for immunohistochemical staining. J Clin Pathol 1999; 52: 75–77.1034361810.1136/jcp.52.1.75PMC501013

